# Physicochemical Characterization of Chitosan-Decorated Finasteride Solid Lipid Nanoparticles for Skin Drug Delivery

**DOI:** 10.1155/2022/7792180

**Published:** 2022-08-06

**Authors:** Muhammad Sohaib, Shefaat Ullah Shah, Kifayat Ullah Shah, Kifayat Ullah Shah, Nauman Rahim Khan, Malik Muhammad Irfan, Zahid Rasul Niazi, Abdulsalam A. Alqahtani, Ali Alasiri, Ismail A. Walbi, Sajid Mahmood

**Affiliations:** ^1^SRDDR, GCPS, Faculty of Pharmacy, Gomal University, D.I. Khan, Pakistan; ^2^Faculty of Pharmacy, Gomal University, D.I. Khan, Pakistan; ^3^Department of Pharmacy, Quaid-i-Azam University, Islamabad, Pakistan; ^4^PDDDL, GCPS, Faculty of Pharmacy, Gomal University, D.I. Khan, Pakistan; ^5^Department of Pharmacy, KUST, Kohat, Pakistan; ^6^Department of Pharmaceutics, College of Pharmacy, Najran University, Najran, Saudi Arabia; ^7^Department of Clinical Pharmacy, College of Pharmacy, Najran University, Najran, Saudi Arabia

## Abstract

Finasteride is considered the drug of choice for androgenic alopecia and benign prostate hyperplasia. The aim of the study was to formulate nanodrug carriers of finasteride with enhanced retentive properties in the skin. The finasteride was formulated as solid lipid nanoparticles that were decorated with different concentrations of chitosan for improved retentive properties. Solid lipid nanoparticles (SLNs) were synthesized by “high-speed homogenization technique” using stearic acid as a solid lipid while PEG-6000 and Tween-80 were used as surfactants. The SLNs were evaluated for particle size, polydispersity index (PDI), zeta potential, drug entrapment efficiency, and drug release behavior. The mean particle size of SLNs was in the range of 10.10 nm to 144.2 nm. The PDI ranged from 0.244 to 0.412 while zeta potential was in the range of 8.9 mV to 62.6 mV. The drug entrapment efficiency in chitosan undecorated formulations was 48.3% while an increase in drug entrapment was observed in chitosan-decorated formulations (51.1% to 62%). The *in vitro* drug release studies of SLNs showed an extended drug release for 24 hours after 4 hours of initial burst release. The extended drug release was observed in chitosan-coated SLNs in comparison with uncoated nanoparticles. The permeation and retention study revealed higher retention of drug in the skin and low permeation with chitosan-decorated SLNs that ranged from 39.4 *μ*g/cm^2^ to 13.2 *μ*g/cm^2^. TEM images depicted spherical shape of SLNs. The stability study confirmed stable formulations in temperature range of 5°C and 40°C for three months. It is concluded from this study that the SLNs of finasteride were successfully formulated and chitosan decoration enhanced the drug retention in the skin layers. Therefore, these formulations could be used in androgenic alopecia and benign prostate hyperplasia to avoid the side effects, drug degradation, and prolonged use of drug with conventional oral therapy.

## 1. Introduction

Finasteride is a competitive inhibitor of 5-*α*-reductase (type-II), commonly prescribed for the treatment of benign prostate hyperplasia (BPH) and male pattern baldness (androgenic alopecia). Both the disorders occur due to the high level of testosterone conversion into more potent form, i.e., dihydrotestosterone, by the action of 5-*α*-reductase. Dihydrotestosterone cause rapid growth of prostate tissue and destruction of hair follicles [1]. Finasteride competitively blocks the action of 5-*α*-reductase and hence can be used in the treatment of these diseases. According to BCS, finasteride is classified as class II drug which possesses high permeability and low solubility that directly affects the dissolution and bioavailability of the drug [2, 3]. The approved daily dose of finasteride in androgenic alopecia is 1 mg/day, and for BPH, it is 5 mg/day. It takes months to achieve the desired drug effects because of low drug solubility which may cause side effects in the form of gynecomastia, mood disturbances, and sexual problems, i.e., decreased libido and erectile and ejaculation disorders [4, 5].

Natural polymers have been extensively used in drug formulations because of their nontoxic, biocompatible, and biodegradable nature. Chitosan is a natural cationic polysaccharide, obtained from alkaline deacetylation of natural chitin which is extensively present in the exoskeletons of fungal cell wall, arthropods, and crustacean shells [6]. Chitosan promotes dermal absorption of drugs by bioadhesion and opening of the intracellular junctions to allow the entry of polar drugs. This effect of chitosan is most likely due to the positive charge of its amino groups, which provides a strong electrostatic interaction with negative charge on the surface of dermal cells and other molecules such as nucleic acids [7].

Topical/transdermal drug delivery is an alternative and effective route of drug administration because it avoids systemically produced side effects, first pass metabolism, and poor patient compliance. Nowadays, many formulations have been developed to produce local therapeutic effects [8, 9]. For maximum drug absorption through skin, various techniques are investigated and developed such as electroporation, iontophoresis, microneedles, ultrasounds, and microwave treatment, and the most recently nanodrug carriers have led to major interest in the transdermal drug delivery system [10].

The nanocarriers such as nanoemulsions, vesicular drug carriers, and lipid nanoparticles have several advantages in pharmaceutical and cosmetic applications over the conventional dosage forms [11]. Among these carriers, SLNs have gained most interest due to the smallest particle size, improved physical stability, low toxicity, low chemical degradation, flexibility in modulated drug release, less side effects, and low production cost [12, 13]. The use of solid lipid also provides an additional advantage of uniform particle size, increased surface area, and drug loading. The lipids used in SLNs are physiological lipids having similar physiological properties to those of the lipids of the skin, and so these lipids enhance cellular interactions resulting in an improved permeability. Due to this reason, SLNs are considered the most suitable drug carrier for topical, dermal, and transdermal drug deliveries [14]. A number of formulation techniques have been designed to prepare SLNs, among them high speed homogenization and microemulsion techniques are most commonly used. In the preparation, molten solid lipid is mixed with the aqueous surfactant solution followed by homogenization at high pressure. The subsequent cooling of the mixture resolidifies the lipid resulting in SLN formation [15]. The size of the SLNs used for skin drug delivery usually ranges from 1 nm to 1000 nm. SLNs increase the skin permeation, drug solubilisation, and retention of drug into the skin layers by fluidizing the stratum corneum [16]. Various researchers have been working on SLNs to enhance the solubility and bioavailability of drugs by delivering nanoparticulate drugs in modified tablets, microspheres, microemulsions, and transdermal patches [17, 18].

The aim of the present work was to improve the bioavailability of finasteride by formulating it as SLNs with enhanced drug retention properties for topical use. Finasteride drug delivery through skin reduces its major systemic side effects due to its oral administration and could improve drug penetration and accumulation in the layer of skin and hair follicles [12, 19, 20].

## 2. Materials and Methods

Finasteride was gifted by Ferozson's Pharmaceutical Laboratories, Pakistan. Stearic acid, chitosan (low molecular weight), PEG-6000, and Tween-80 were purchased from Sigma-Aldrich®, USA. Healthy male Sprague-Dawley rats were purchased from the University of Peshawar, Pakistan. All the chemicals used in the research were of analytical grade and used without any further purification.

### 2.1. Preparation of Finasteride SLNs

SLN formulations were prepared by a high-speed homogenization method [21]. In these formulations, stearic acid was used as a solid lipid, Tween-80 as surfactant, and PEG-6000 as cosurfactant. The formulation was prepared by mixing the aqueous phase containing an emulsifier with the lipid phase containing a known quantity of active drug. The aqueous phase was prepared by adding Tween-80 and PEG-6000 into a known quantity of distilled water with constant stirring on a hot plate magnetic stirrer, and the temperature was maintained at 75°C. The lipid phase was prepared by melting stearic acid at 75°C and mixing of finasteride in it. The aqueous phase was dropwise mixed with the lipid phase at the same temperature of both phases, i.e., 75°C with constant stirring for one hour. The emulsion was then subjected to homogenization for 7 minutes at 10,000 rpm. The final formulation was then immediately cooled at 10°C using an ice bath to obtain SLNs. Chitosan was added to the water phase with different ratios (0.125%, 0.25%, 0.5%, and 1%). Chitosan was solubilized in 1% acetic acid solution and incorporated into the aqueous phase containing surfactants (Table 1).

## 3. Physicochemical Characterization

### 3.1. Particle Size, Polydispersity Index, and Zeta Potential

Particle size has a prime importance in bioavailability and therapeutic index [22]. The samples were evaluated for particle size, polydispersity index (PDI), and zeta potential by photon correlation spectroscopy using Zetasizer (ZS90 Zetasizer; Malvern Instruments Ltd., Worcestershire, UK) at room temperature. For analysis, 5 mg of SLNs was diluted in 5 ml of deionized water and analyzed on Zetasizer. All the experiments were performed in triplicate [23].

### 3.2. Entrapment Efficiency

The drug entrapment efficiency (E.E) was determined to check the concentration of free drug in the dispersion medium [24]. Briefly, 1 ml of dispersion was diluted with 4 ml of distilled water, and the mixture was centrifuged at 15000 rpm for 30 minutes. The supernatant layer was collected and checked for drug contents through HPLC at *λ* max of 210 nm.

E.E was measured by the following formula:

(1) $$\begin{array}{c} \text{E}.\text{E}=\left(\frac{W_{\text{T}}-W_{\text{F}}}{W_{\text{T}}}\right)\times 100\%, \end{array}$$

where E.E is the entrapment efficiency of SLNs, *W*_T_ is the total weight of finasteride added at the time of preparation, and *W*_F_ is the weight unloaded finasteride filtered in the supernatant layer.

### 3.3. Infrared Spectroscopy (ATR-FTIR)

All the formulations were subjected to Fourier transform infrared (ATR-FTIR) spectroscopy to check any possible interactions of the formulation components. For this purpose, samples were analyzed as liquid suspension of SLNs and the spectra of ATR-FTIR were taken within the frequency range of 400 to 4000 cm^−1^ and ambient air as a background, using FTIR spectrophotometer (PerkinElmer Inc., Waltham, MA, USA) while the peaks were determined using Perkin Elmer Spectrum version 6.0.2 software (PerkinElmer, Waltham, MA, USA) [25].

### 3.4. *In Vitro* Drug Release Studies

The drug release studies were performed on the Franz diffusion cell (PermeGear, USA) with little modification in the already reported method [26]. For this, the receptor compartment was filled with 6 ml of acetate buffer solution pH 5.5 (USP) in simulation of skin, and the donor compartment was loaded with 3 ml of SLN sample. An artificial membrane (polytetrafluoroethylene (PTFE), 0.45 *μ*m pore size; Sartorius AG, Goettingen, Germany) were mounted in between the donor and receptor compartments. The temperature of the receptor compartment was maintained at 32 ± 2°C. The buffer solution in the receptor compartment was magnetically stirred at 200 rpm throughout the study [27]. The study was performed for 24 hours, and with the help of a sterilized syringe, 0.5 ml of aliquots was withdrawn from the receptor compartment with the time intervals of 0, 0.5, 1, 2, 4, 8, 12, 16, and 24 hours for further analysis and the same amount of fresh buffer was added to maintain the volume. The samples were then analyzed using HPLC for drug contents.

### 3.5. *Ex Vivo* Drug Permeation Studies

*Ex vivo* drug permeation studies were performed on healthy male adult Sprague-Dawley rats having weight 220 g ± 10 [28]. For this, after the approval of the ethical review committee via notification no. 823/QEC/GU dated 18/06/2019, rats were divided into 5 groups each containing 3 rats (*n* = 3/formulation). The rats were anesthetized using injections of ketamine and xylazine in the doses of 15 mg and 2 g, respectively, per 220 g of the body weight of rats. The skin was shaved from the back of rats using a sterilized razor. The rats were euthanized by cervical dislocation, and the skin was extracted from the back side, washed with normal saline, and kept in a freezer at -40°C till used. The skin was thawed and cut into pieces as per size of the donor compartment of Franz diffusion cell. The receiver chamber was filled with the phosphate buffer solution (pH 7.4). The skin was mounted between the donor and receptor chamber in such a way that its epidermis was in direct contact with the formulation, i.e., facing towards the donor chamber. The temperature of the Franz diffusion cells was maintained at about 37°C ± 2, and the formulations were poured into the donor chamber. The samples were drawn after the time intervals of 0, 0.5, 1, 2, 4, 8, 12, 16, and 24 hours. The same amount of fresh buffer was replaced in the receiver chamber every time after the samples were withdrawn, to maintain the constant amount of buffer solution in the receiving chamber. The samples were then evaluated through HPLC for drug contents. The cumulative amount of drug permeated was then plotted against time.

## 4. Results and Discussion

### 4.1. Particle Size Distribution and Zeta Potential

The particle size distribution and surface charge are determined to predict the therapeutic performance and stability [29]. The particle size, PDI, and zeta potential of the freshly prepared SLNs are shown in Table 2. The particle size of blank SNLs (F0) was 10.10 ± 1.046 nm, comparatively smaller than all other formulations. Incorporation of the drug into the formulations increased the particle size (F1) being 14.68 ± 1.841 nm. The smallest particle size of the SLNs might be due to the addition of surfactants in the formulations which reduced the surface tension resulting in the smallest particle size [30]. It was observed that the particle size of the drug-loaded SLNs (F1-F5) was greater than that of the blank (F0) which depicts the successful encapsulation of drug in the solid lipid formulation that increased the particle size [31]. Chitosan coating further increased the particle size and zeta potential in formulations (F2-F5) which was due to the deposition of chitosan layers over the SLNs. Higher concentration of chitosan caused more increase in particle size suggesting the thicker layer formation due to the stronger interaction of stearic acid and positively charged chitosan. The inversion of positive charge may be because of amine group of chitosan [32–34]. No further increase in PDI values was observed which was likely due to the increased repulsive forces among the positively charged surfaces of the SLNs [35, 36]. Increase in zeta potential values was observed with increase in the concentration of chitosan indicating the formation of thicker layer of chitosan over the SLNs which increased the positive surface charge due to the protonated aliphatic amino groups of chitosan which gave it a cationic nature, so addition of chitosan inverts the negative charge to positive and increase in concentration increases the positive charge [37].

### 4.2. Entrapment Efficiency

Drug entrapment efficiency (E.E) and drug association efficiency (DAE) were checked as per previously explained methods with few modifications [24].

The E.E results showed successful encapsulation of the drug within SLNs for both undecorated (48.3% ± 1.6 for F1) and chitosan-decorated formulations (51.1% ± 2.2, 54.2% ± 2.4, 57.1% ± 2.9, and 62% ± 3.3 for F2-F5). The low percentage of drug entrapment was due to the crystallinity of solid lipid used which was also reported in the previous studies [38]. The selection and amount of lipid affect the E.E; solid lipids have less solubility of drugs than liquid lipids because they possess higher melting points and have crystalline nature at room temperature. Similarly, more amount of lipid encapsulates more drug and vice versa [39, 40]. So finasteride-loaded stearic acid SLNs are having more capacity of drug loading which makes them safer for use. Similar types of results were also discussed in the previous study where the SLNs of stearic acid showed drug entrapment of 68.38% [41].

### 4.3. Fourier Transform Infrared Spectroscopy (FTIR)

The FTIR spectra (Figure 1) show the results of pure drug as well as the components of the formulation and polymer. In the spectra of pure finasteride, absorption bands at 1600 to 1666 cm^−1^ are of amide groups while at 2917 cm^−1^, they are of C-H stretch. Other band peaks at 1390-1400 cm^−1^ are of tertiary butyl group in finasteride.

Mixing of finasteride with other components of the formulation as well as the polymer (chitosan), in physical form and after developed optimized SLN formulation, did not show any interaction, and hence, no interference was observed with the characteristic drug peaks which confirms the compatibility of drug with the additives, as mentioned previously [42, 43]. Stearic acid spectra in Figure 1 show a carbonyl peak at 1697.51 while peaks at 2848.04 and 2915.09 are recognized as CH2 symmetric stretch and CH2 antisymmetric stretch. The same peaks were also reported by Singh et al. in a study [44]. Chitosan spectra have peaks at 1667.1 cm^−1^ which shows the amine group and 2917.74 cm^−1^ which shows C–H stretching and a distinctive wide band at 3439.2 cm^−1^ which is due to OH/NH_2_ stretching vibrations [45–47].

### 4.4. Transmission Electron Microscopy

Transmission electron micrographs (Figure 2) also confirmed the monomolecular nanoparticle size of the SLNs in the formulations. The images showed increase in the particle size with the increasing concentration of chitosan while no intraparticle interaction was observed. TEM images demonstrated the nanosize and uniform distribution of the SLNs while the influence of chitosan coating in an increase in the particle size was also observed which was due to the formation of chitosan layers over the particles [48, 49].

### 4.5. *In Vitro* Drug Release Studies

In *in vitro* drug release study, as explained in Figure 3, all the formulations showed a sustained release pattern except F1 that showed an initial burst release of finasteride due to small particle size and no polymer decoration that can hinder drug release from formulations. The complete drug was released within 12 h. In the case of F2 to F5, the drug release was sustained due to the addition of chitosan, and even after 24 hours, only 60% of the drug was released [50]. Previous studies also showed slow release of drug from chitosan-coated SLNs after 24 hours (60% to 90%) which was supposed to be due to the deposition of particles in the superficial layers of skin and swollen nature of chitosan in hydrophilic environment [23, 51, 52].

The SLNs possess slower polymorphic transition of stearic acid, so the solid lipid in the formulation gives more stable formulation. The vesicles mostly remain in amorphous form, thereby favouring formation of pores and easy solvation of drug in nanoparticles [53]. Generally, the pressure will cause some detectable changes in hydration because it induces changes in ionization of surface charges due to either electrostriction or changes in charge repulsion, so the particles remain separated from each other for longer period of time which enhances the stability of the formulation. However, the individual stable particles can be penetrated easily by dissolution medium, thereby favouring initial burst release [54]. Chitosan being cationic polymer coats the vesicles of SLNs that control the release of drug from the nanoparticles that follow nonfickian diffusion when determined using the Korsmeyer-Peppas equation. Similarly, regarding membrane-polymer interactions, the amino group of chitosan had been shown to improve the muco-/bioadhesive properties enabling ions to go through so-called ion channels [55].

### 4.6. Permeation and Retention Study

The permeation of drug through intact skin depicted significantly higher permeation for nondecorated SLNs (F1) in comparison to its coated counterparts (F2-F5). This was due to the lipoidal interaction of skin with solid lipid of the formulations. Furthermore, the presence of surfactants further potentiates penetration of drug through the skin. The permeation of 42.7% was achieved for F1 that gradually reduced to 12.8% in the case of F5 (Figure 4). The relatively lower permeation in the case of chitosan-coated formulations could be attributed to larger particle size and high viscosity of the coated SLNs [56]. The findings of permeation study signify the importance of physicochemical properties of SLNs in improved permeation of drug through the skin.

The retention of drug in intact skin from SLNs delivered topically has shown that chitosan-decorated SLNs achieved significantly higher drug retention due to bioadhesive properties of chitosan [57]. The retention of drug increased linearly with increasing concentration of chitosan in SLNs (Figure 5). The cationic nature of chitosan that interacted with the negatively charged skin layers could also be the prominent feature in higher drug retention from formulations (F2-F5) as revealed in the previous studies [58–62].

### 4.7. Stability Study

All the formulations were evaluated for their stability for 3 months at 05 ± 2°C and 40 ± 2°C [63]. The stability was checked by evaluating the mean particle size, zeta potential, pH, and viscosity [64]. The results have shown no phase separation and no significant change in the pH and zeta potential, but a slight increase in particle size and viscosity was observed which was due to the sedimentation of particles and evaporation of water (Figure 6). On storage, the solid lipid gives more stable formulation because it possesses slower polymorphic transition of hydrocarbons [65].

## 5. Conclusion

The finasteride-loaded chitosan-coated SLNs were successfully prepared by a high-speed homogenization method from physiologically inert substances. Stearic acid was used as a solid lipid in the formulations. On the basis of obtained results in terms of particle size, PDI, zeta potential, pH, and E.E, developed formulations could be used for application on the skin. The SLNs have shown excellent compatibility and no interaction among the ingredients as revealed by FTIR. *In vitro* release indicated the burst release without chitosan coating while slow sustained release pattern was observed in the case of chitosan-coated SLNs. Higher permeation was observed with chitosan-uncoated SLNs as compared to chitosan-coated SLNs. Moreover, chitosan coating also significantly enhanced the retention of drug within the skin layers. Based on these findings, it was concluded that chitosan-coated SLNs could be used as an alternative to oral drug delivery of finasteride in androgenic alopecia and benign prostate hyperplasia to overcome the harmful side effects and patient compliance.

## Figures and Tables

**Figure 1:** FTIR of finasteride: formulation and its components.

**Figure 2:** Transmission electron microscopy of SLNs.

**Figure 3:** *In vitro* drug release profile of SLNs through intact skin.

**Figure 4:** Permeation of drug through intact skin from SLNs.

**Figure 5:** Retention of drug from SLNs in the intact skin.

**Figure 6:** Stability studies of SLNs.

**Table 1:** Formulation composition (finasteride, chitosan, stearic acid, and Tween-80) of SLNs.

F. code	Drug (% *w*/*w*)	Stearic acid (% *w*/*w*)	PEG-6000 (% *w*/*w*)	Tween-80 (% *w*/*w*)	Chitosan (% *w*/*w*)	Acetic acid (% *w*/*w*)	Water (% *w*/*w*)
F0	—	1.5	1	2.5	—	—	95.000
F1	0.1	1.5	1	2.5	—	—	94.900
F2	0.1	1.5	1	2.5	0.125	28.108	66.667
F3	0.1	1.5	1	2.5	0.250	41.316	53.334
F4	0.1	1.5	1	2.5	0.500	61.065	33.335
F5	0.1	1.5	1	2.5	1.000	73.900	20.000

**Table 2:** Effect of chitosan coating on particle size, PDI, pH, and viscosity of SLNs.

Formulation code	Particle size (nm)	PDI	Zeta potential (mV)	pH	Viscosity (cp)
F0	10.10 ± 1.046	0.412 ± 0.012	8.9 ± 6.23	5.3 ± 0.652	3.0 ± 0.8
F1	14.68 ± 1.841	0.369 ± 0.043	18.7 ± 8.80	5.5 ± 0.841	3.5 ± 1.1
F2	76.74 ± 2.122	0.297 ± 0.004	23.5 ± 5.59	5.6 ± 0.893	4.5 ± 2.3
F3	109.6 ± 4.363	0.244 ± 0.027	32.1 ± 7.09	5.6 ± 0.789	5.5 ± 2.8
F4	122.4 ± 5.214	0.313 ± 0.016	50.8 ± 8.73	5.5 ± 0.854	23.3 ± 5.6
F5	144.2 ± 6.931	0.291 ± 0.019	62.6 ± 7.98	5.5 ± 0.968	170 ± 18.4

## Data Availability

The data used to support the findings of this study are included within the article.
